The article "Microencapsulation of Fe2+ in Spray-Dried Lactose for Improved Bioavailability" was retracted in 2023. Reasons: signs of a paper mill; compromised peer review; unreliable results or conclusions.

# Microencapsulation of Fe2+ in Spray-Dried Lactose for Improved Bioavailability

**DOI:** 10.1155/2021/5840852

**Published:** 2021-09-15

**Authors:** Nan Li, Xu Li, Ping Yang, Hongbin Liu, Lingyu Kong, Xiaomeng Yu

**Affiliations:** ^1^Pharmaceutical Analysis Center of Tianjin Institute of Medical and Pharmaceutical Sciences, 79 Duolun Road, Heping District, Tianjin 300020, China; ^2^Cardiovascular and Cerebrovascular Drugs Research and Development Center of Tianjin Institute of Medical and Pharmaceutical Sciences, 79 Duolun Road,Heping District, Tianjin 300020, China; ^3^Tianjin Institute of Medical and Pharmaceutical Sciences, 79 Duolun Road, Heping District, Tianjin 300020, China; ^4^Experimental Animal Center of Tianjin Institute of Medical and Pharmaceutical Sciences, 2 Wanquan Road, Hepign District, Tianjin 300020, China

## Abstract

The development of spray drying technology has been widely used for drying and preservation of food products. Though infant milk powder iron fortification is necessary for infants and children, iron fortification is accompanied by some limitations that reduce its quality and oxidation of Fe2+ into Fe3+, causing sensory problems and even a decrease in iron absorption, which does not meet the normal requirements of infant and child body development. To overcome this adverse effect and to improve the bioavailability of iron, a spray drying method was used to simulate the milk powder production process by codrying a mixture of ascorbic acid and ferrous sulfate, where ascorbic acid was uniformly coated on the outer layer of ferrous sulfate. It was demonstrated that ascorbic acid had a very obvious inhibitory effect on the oxidation of ferrous iron and could maintain the stability of ferrous iron in solid and solution for a long time, thus improving the bioavailability of iron.

## 1. Introduction

Iron is an essential element for living organisms, and its ability to convert between trivalent and divalent iron makes it essential for many biochemical functions such as energy production, DNA synthesis, and oxygen transport, which are particularly important for the energy metabolism, brain development, immune function, and thermoregulation in the body. Iron deficiency, especially during the rapid growth and development of infancy, can have serious and sometimes irreversible effects on long-term health. At this time, iron deficiency interferes with the normal function of neurotransmitters, causing delayed brain development in infants and children, resulting in cognitive and psychomotor developmental deficits that can be lifelong despite subsequent correction of iron deficiency [1–3]. Therefore, it is critical that nursing infants have enough iron to meet their developmental needs. In many studies, scientists have cited the adverse effects of iron deficiency on infant and child growth and development. Under normal physiological conditions, iron enters the body in large quantities from only two sources: across the placenta during fetal life and through the wall of the small intestine after delivery. In addition to iron stores at birth, infants also receive iron from their diet, which often includes breast milk or other iron-containing fortifications [4]. However, this iron is utilized very rapidly during the first few months of life, and during the second half of infancy, the continued rapid growth and expansion of hemoglobin mass and the depletion of iron stores result in high iron requirements for infants [5–7]. Despite the high bioavailability of iron in human milk, the concentration of 0.20–0.35 mg/L of iron in human milk is very low, and thereafter, dietary iron becomes the primary source for humans [8, 9]. The American Academy of Pediatrics (AAP) recommends that infants at 6 months of age should consume iron-fortified infant cereals and supplements [10–12]. Iron supplementation during infancy and childhood can be achieved in different ways, including foods high in iron, direct administration of supplements, or iron fortification of certain dairy products. Although these methods are simple, the high cost and low bioavailability hinder the rationality of their application. Moreover, the application of iron in dairy products can easily cause color, taste, odor, or texture deviations due to the conversion of the free ferrous state (Fe2+) to the trivalent iron state (Fe3+). This can cause serious side effects in children, including discoloration of teeth, nausea, vomiting, black stools, and diarrhea. Therefore, preventing the oxidation of ferrous iron (Fe2+) to trivalent iron (Fe3+) in iron-fortified foods is an important way to increase the stability of iron in foods and improve the efficiency of iron supplementation during infancy and adult [13, 14].

Vitamins are also organic compounds designated as nutrients, a class of substances that cannot be synthesized in the human body on its own and can only be obtained through food [15]. Water-soluble ascorbic acid (AA) is one of them, and its deficiency in the body induces many undesirable diseases. The most iconic disease caused by AA deficiency is scurvy, which occurs mainly due to abnormalities in collagen synthesis caused by abnormal hydroxylation of proline and lysine. This compound reacts with various free radicals, is widely present in cells, and is considered a perfect antioxidant for almost all oxygen-demanding biological cells [16]. AA has also been shown to increase the absorption of iron in the body [17, 18]. Using AA to reduce or even avoid Fe3+ in food fortification seems to be a perfect choice.

In this experiment, the encapsulation of Fe3+ by AA was accomplished by the spray drying technique. Spray drying is one of the most popular, simple, economical, and common encapsulation techniques [19]. The feed material enters the atomizer through the feed pump, which decomposes the liquid feed into small droplets and introduces them into the drying chamber, and the atomized droplets are instantly dried by contacting with hot gas. At the same time, the heating gas can be replaced with nitrogen in order to prevent oxidation of the material inside the droplets. The dried particles are separated from the drying air and collected in the bottom of the vessel [19, 20]. In this method, the encapsulation ratio of product size and shape is controlled, and the operation is simple and economical for the encapsulation of ferrous sulfate.

## 2. Materials

We chose ferrous sulfate heptahydrate ( > 99.0%) as the provider of divalent iron. It was purchased from Zhiyuan Chemical Reagents Co., Ltd., Tianjin. Ascorbic acid (99.7%) was purchased from Xilong Scientific Co., Ltd. The pharmaceutical grade *α*-lactose monohydrate (purity ≥ 99.9%) was provided by Jiangsu Dawning Pharmaceutical Co., Ltd., China. The purified water used in this experiment was made in laboratory.

## 3. Experimental Design

In order to mix ferrous sulfate and ascorbic acid as much as possible at the molecular level or to make ferrous sulfate as wrapped as much as possible by ascorbic acid, we codissolved them in pure water. Since both ferrous sulfate and ascorbic acid are highly soluble in water, we made our own pure water as the dispersion medium for both substances in our experiments. This was done by dissolving a prescribed amount of AA in 200 ml of water, as expected, and then dissolving 1.0 g of ferrous sulfate in the above solution. To exclude the influence of the manipulation process on the results, a pure ferrous sulfate solution was prepared. Interestingly, but the instant ferrous sulfate was dissolved in water, the color of the solution was no longer transparent, gradually appeared yellow, and the color deepened, and a tan precipitate appeared after standing, while the solution of ferrous sulfate with AA added remained transparent.

The experiment was started, and the molar ratios of ferrous sulfate and AA were obtained as 1 : 1, 2 : 1, 5 : 1, and the solution/mix without the addition of AA, respectively. The solutions/suspensions were fed at the same feed rate under stirring. The same spray drying parameters were used for both suspensions, and the spray dryer (Shanghai YC-015) was adjusted to the optimum parameters as follows: fan frequency 50.0 Hz, inlet air temperature 130°C, outlet air temperature 120°C, peristaltic pump speed 18.0 ml/min, spray pressure 0.25 MPa, and nozzle diameter 1.0 mm. Each sample solution/suspension was spray-dried separately, respectively, the powder samples *A*, *B*, *C*, and *D* were obtained.

## 4. Characterization of Samples

### 4.1. UV-Visible Spectrophotometer (UV-Vis)

The resulting sample powders were configured according to the iron content, and each sample was dissolved in water at 70°C and cooled to room temperature separately. The aqueous solutions were individually configured, so that the iron content in each solution was consistent. Based on the wavelength theory for detection of absorption maxima of ferrous ion compounds proposed by Tomáš Filipský in 2013, we detected absorption at wavelengths 200–500 nm due to the properties of absorption spectra [21]. The instrument used is the UV-2401 PC spectrophotometer, Shimadzu, Kyoto, Japan.

### 4.2. Differential Scanning Calorimetry (DSC)

The obtained sample powders were analyzed by DSC using a differential scanning calorimeter (HSC-4 DSC, Henven, China). Samples for DSC determination were prepared using a sealed aluminum pan following standard procedures. Approximately 6.0 mg of each specimen was used in the analysis.

### 4.3. Fourier Transform Infrared Spectroscopy (FTIR)

The raw materials and samples were studied using Fourier transform infrared spectroscopy (FTIR). The samples were compounded with dried KBr powder, pressed into transparent sheets, and scanned for transmission sensitivity in a Nicolet 6700 FTIR spectrometer (Thermo Fisher Scientific). The resolution of the FTIR spectrum was 1 cm^−1^.

### 4.4. Scanning Electron Microscope (SEM)

The sample was placed on an aluminum sample peg with a carbon tape. The gold-plated samples were examined with a JSM-7200F scanning electron microscope (SEM, JEOL Ltd.).

### 4.5. Thermo Gravimetric Analyzer (TGA)

The samples were analyzed using a thermo gravimetric analyzer (TGA Q5000 V3.17 Build 265). The samples were tested in an alumina pot with N2 as equilibrium gas. The temperature was set at 40°C–350°C, and the heating rate was 5°C/min.

### 4.6. N_2_ Absorption

Separate N2 adsorption experiments were performed on powder samples to evaluate the difference in porosity of different samples.

### 4.7. X-Ray Diffraction (XRD)

The sample powders were studied by the XRD analysis by a Siemens D5000 diffractometer.

## 5. Results and Discussion

By direct observation of the color of the solution (Figure 1), we can see that the solution without the addition of ascorbic acid has a very distinct tan color, and the color is darker after spraying high temperature and high humidity environment. For the two samples with added AA, the low percentage was slightly yellow and the high percentage was completely transparent in the solvent. Ferrous ions form chelates with ascorbic acid, and maximum absorption is found at 266 nm (Figure 2) after spray drying. No absorption peak at 266 nm was found for the physical mixture without AA addition and spray-dried sample A without AA addition. The overall absorption of spray sample *A* was relatively weak after dissolution and high temperature treatment, showing the catalytic ability of high temperature and humid environment on ferrous iron oxidation. Sample *B* (Fe2+ : AA = 5 : 1(m/m)) showed a weak absorption at this position, which indicates that AA has a protective effect on ferrous ions in a high temperature and humid environment. Strong absorption was observed for sample *C* (2 : 1(m/m)) and sample *D* (1 : 1(m/m)), with a higher ratio of AA having a stronger protective effect on ferrous ions. The absorption of sample *D* and sample *C* is essentially the same, which may be due to two reasons; one is because all the ferrous ions in sample *D* are chelated with AA in the form of Fe2+ and the excess AA pure substance does not increase the absorption intensity; the second may be because there is almost no difference in the protective effect of the two ratios of AA on Fe2+.

The change in peak intensity or wave number shift was studied by FTIR (Figure 3). For ferrous sulfate heptahydrate, only absorption peaks of crystalline water appeared in the tested interval. Absorption peaks for each raw material were observed in the physical mixture. However, for the spray-dried sample, each sharp absorption peak disappears and a gentle blunt absorption peak appears, suggesting the appearance of amorphous products. This indicates a decrease in the density and strength of hydrogen bonds and a decrease in crystalline states. The absorption peaks and trends of the spray products were basically the same, but the characteristic peak of AA appeared in sample *C* at 1754 cm^−1^, which suggested that some AA might not be chelated with ferrous ions.

We performed thermal analysis of each raw material and spray-dried samples. By analyzing the DSC curves of the samples (Figure 4), the heat absorption peaks of lactose appeared at 148°C and 209°C for its crystalline water and lactose crystals, respectively, the heat absorption peak of AA appeared at 196°C for Tim; the heat absorption peak of crystalline water of ferrous sulfate heptahydrate appeared in the physical mixture during the heating process, the crystalline water peak moved to the high temperature region at 148°C, and the heat absorption peaks of AA and lactose crystals broadened and combined together. However, for the spray-dried sample, multiple free water and crystal water heat absorption peaks appeared, suggesting a complex chelation structure. According to TGA (Figure 5) curves, the weight loss trends of multiple samples were basically similar in the same temperature range. The difference is that the weight loss trend of sample B is steeper at each temperature, and the sample may have less by-products.

By comparing the sample XRD patterns (Figure 6) with the available literature XRD patterns, any phase change in the raw material was ruled out. The new reflections observed in the cocrystal pattern can be attributed to the formation of cocrystals formed by the combination of ascorbic acid and lactose and ferrous sulfate. The present data are insufficient to indicate the crystal system of the formed cocrystals. The position and size of the curved peaks in all three samples are essentially the same, suggesting the formation of identical cocrystals. Sample *B* was less intense and had a flatter peak shape compared to samples *A* and *B*, probably due to the formation of more amorphous solid products.

We also observed the scanning electron microscope (Figure 7), and the 5000x and 2000x fields of view of the three typical samples are placed in figure. We can see the porous structure of the sample surface with smooth surface inlaid with the crystalline material. The SEM fields of the three samples have very little difference at the same magnification. We have observed the existence of pore structures in each sample in SEM. Through the combined analysis of the BET and BJH (Figure 8) data, we found that the internal pore structure of each sample is basically the same. By the combined analysis, the average pore size of the samples is between 7.6 and 8.4 nm, which has a large internal pore volume (BJH desorption cumulative volume of pores between 1.7000 nm and 300.0000 nm; width: 0.088348 cm^3^/g) and pore surface area (BET surface area: 38.9802 m^2^/g). The pore structure of the ferrous sulfate sample provided its good stability and dissolution rate, which is very favorable for fortification of food applications.

## 6. Conclusion

Supplementation of ferrous iron in fortified foods, especially the ferrous component of the formulation, is particularly necessary. In the present experiment, ferrous sulfate was encapsulated with ascorbic acid and lactose crystals by using ascorbic acid and ferrous sulfate cospray. The results showed that the proper ratio of ascorbic acid has a good antioxidant effect on ferrous sulfate, protects ferrous ions from oxidation in high temperature and high humidity environments, and preserves ferrous iron in food well for optimal supplementation at the time of intake. This has good applications in iron supplementation and in increasing iron absorption through food.

## Figures and Tables

**Figure 1:** Direct observation of the color of the solution.

**Figure 2:** UV absorption curve of each sample at 200–500 nm.

**Figure 3:** Infrared absorption spectrum of each spray-dried sample and raw material.

**Figure 4:** DSC curves of spray-dried samples and raw materials.

**Figure 5:** TGA curve of each spray-dried sample.

**Figure 6:** XRD curves of each spray-dried sample.

**Figure 7:** SEM view of a typical spray-dried sample (*A*1 and *A*2 for sample *A*; *B*1 and *B*2 for sample *B*; *C*1 and *C*2 for sample *C*, respectively.

**Figure 8:** Typical spray-dried sample nitrogen adsorption curve. (a) Isotherm linear plot. (b) BJH adsorption dV/dlog(w) pore volume.

## Data Availability

The data used to support the findings of this study are included within the article.
